The article "Gel scaffolds and emerging applications in biomedicine" was retracted in 2023. Reasons: plagiarized text; overlap with other authors' work.

# Gel scaffolds and emerging applications in biomedicine

**DOI:** 10.1039/d2ra00924b

**Published:** 2022-05-26

**Authors:** Mani Rajasekar, Manivannan Lavanya

**Affiliations:** Centre for Molecular and Nanomedical Sciences, International Research Centre, Sathyabama Institute of Science and Technology (Deemed to be University) Chennai – 600 119 Tamilnadu India drmrajasekar.irc@sathyabama.ac.in mrajasekar_83@yahoo.com +91-44-24503814 +91-9710230530

## Abstract

Nowadays, gels are formed by small molecules self-assembling under the influence of various non-covalent interactions. They can be easily perturbed, which allows for the careful tweaking of their properties. They are kinetically confined, and following production, they usually do not demonstrate time-variable changes in material properties. When exposed to external stimuli such as temperature, pH, light, enzymes, redox, and chemical analytes, such materials may become switchable, leading to the reconfiguration of the gel matrix into a different type of network. The transformations allow gel-to-gel transitions, while the changes in the molecular aggregation result in the alteration of the physical and chemical properties of the gel with time. Here, we discuss various methods used to achieve gel-to-gel transitions by modifying a pre-formed gel material through external perturbation. The dynamic modification of gels allows the construction of an array of gels with various properties from a single material, which eventually extends the limit of application of the gels.

## Abstract 2

Nowadays, gels are formed by small molecules self-assembling under the influence of various non-covalent interactions.

## 1. Introduction

In recent years, gels (1) have been cross-linked to form polymeric networks that can hold a lot of solvent while keeping their solid-state flexibility. These are semi-solid and tough to describe as a gel, but they are simple to recognize as they do not flow when the tube containing the gel is inverted. On a macroscopic scale, they are frequently translucent, stretchy, moist, and soft. Gelling chemicals, which are frequently low-molecular-weight compounds, are used to build a polymeric scaffold.^1,2^ It can be built in a variety of ways, including the physical entanglement of polymer chains, covalent conjugations, and non-covalent molecular interactions like electrostatic interactions, coordination interactions, hydrophobic interactions, host–guest interactions, and hydrogen-bonding interactions, among others. They are created *via* covalent cross-linking and are solid at the microscopic level but non-covalent connections and physical entanglements are more flexible, allowing the gel to perform dynamic activities such as self-healing and stimulus-responsiveness (Fig. 1).^3–5^ Gel systems can be fine-tuned to incorporate chemically and physiologically active moieties. Furthermore, rational gels are designed at the molecular level and with multi-scale architecture control, resulting in significantly better characteristics and functional applications.^6,7^ They are also an important component of the living stuff found in organs and tissues. They may be programmed to replicate the micro-environments of biological tissue. For tissue repair and regeneration, gels are used as scaffolding matrixes in contact lenses and other injectable and implantable biomaterials.^8^ 3D printing technologies, notably gel-based biological cell printing, offer simple and effective techniques for the design and manufacture of complex living objects at many length scales. In ultrasonic diagnostics, as well as electrophysiological assessments of the brain, heart, and muscle, gels have long been employed to connect metallic electrodes and living tissues.^9^ The gel-derived conducting materials are appealing at human–machine interfaces because of their likeness to real living tissues and their capacity to connect electronics, allowing a wide range of applications. They are being developed as stretchable, transparent ionic conductors for wearable devices such as artificial muscles, skins, and axons in this regard.^10^

**Fig. 1:** Schematic representation of self-assembled gelation (1).

Luminescent gels have been extensively used in human–computer interactions, soft robotics, sensors, bioelectronics, and biomedicine.^9^ However, the singularity of the feature within the gels restricts their similar packages in lots of excessive-tech regions because the regions require materials with multiple features. However, gel materials integrating the functions of luminescence and conductivity simultaneously can show both features of luminescence and conduction and in many cases, have unexpected characteristics due to the synergistic effects. The functional versatility allows the material to find applications in high-tech areas, including biosensors and bioelectronics. Consequently, the primarily gel-based luminescent conductive material as an emerging purposeful cloth has many superior characteristics and has recently made high-quality contributions in biosensors and bioelectronics. In this review, we discuss gel-based luminescent materials and their emerging applications in the biomedical field.

## 2. Azobenzene-based gel

A new series of azobenzene–cholesterol organogel compounds (2) with different spacers were designed and synthesized (Fig. 2a). The molecular structures were confirmed by different NMR techniques. The reversible photoresponsive properties of the compounds were investigated by absorption spectroscopy. Their thermal phase behaviors were studied by DSC. The length of the spacer plays a crucial role in the gelation. These are the only ones that can gelate in ethanol, isopropanol, 1-butanol, and the reversible gel–sol transitions were also investigated. To obtain visual insight into the microstructure of the gels, the typical structures of the xerogels were studied by SEM. The morphologies of the aggregates changed between flower-like, networks, and rods with different sizes. It was found that intermolecular H-bonding, the solvents, and van der Waals interaction are the main contributors to the specific superstructure.^11^ Moreover, the supramolecular gel of the azobenzene-based phenylalanine derivative (3, AZO-Phe) application in methylene blue (MB) adsorption has been developed. The gelator has shown great ability to form stable gels with a critical gelation concentration as low as 1.0 mg mL^−1^ in EtOH/H_2_O. It also showed that the gel has a good adsorptive performance toward MB in aqueous solution. The adsorption process and mechanism of MB on the AZO-Phe gel were systematically investigated. Batch experiments were performed to study the effects of initial dye concentration, contact time, and pH on the adsorption performance of AZO-Phe gel. The adsorption process and data were fitted well with the Langmuir isotherm model and pseudo-second-order kinetic model. Moreover, the AZO-Phe gelator could be recovered after MB adsorption, and the rate of recovery was achieved at 95%. These results provide a mixed solvent gel method for the purification of dye-polluted water systems (Fig. 2b).^12^

**Fig. 2:** (a) The structure of photoresponsive cholesterol-based azobenzene organogels (2). (b) Self-assembly of the azobenzene-based phenylalanine derivative (3).

A phase-selective low-molecular-weight photoswitchable sugar hybrid (4) was synthesized, and the selective gelation of aromatic solvents in a mixture was observed even at micromolar concentrations.^13–15^ The morphological investigation implied the formation of self-assembled fibrillar networks that upon irradiation get chopped into short fibers, affecting the gel–sol transition. The gelator is selective for aromatic solvents that allow the removal of such solvents from an aqueous layer. Such phase-selective photoresponsive gelators may be useful for the removal of small amounts of toxic aromatic solvents from contaminated water (Fig. 3a). In addition, the supramolecular assembly of azobenzene-based biscalix[4]arene (5) was generated in ethyl acetate by laser trapping. The nucleation and growth were elucidated. No trapping behavior was observed when a 1064 nm laser beam was focused inside the solution; however, interesting assembly phenomena were induced when it was shone at the air/solution interface. A single disk having two layers was first prepared at the focal point of ∼1 μm and then expanded to the size of a few tens of μm, although no optical force was exerted outside the focal volume. Upon switching off the trapping laser, needles were generated at the outer layer of the assembly, giving a stable sea urchin-like morphology to the generated assembly. At 30–50% dilution of the initial solution in ethyl acetate, a mushroom-like morphology was also observed. Laser trapping-induced assembly of azobenzene-based biscalix[4]arene was quite different from the sharp ellipsoidal aggregates obtained by the spontaneous evaporation of the solution. These trapping phenomena were specifically observed for the biscalix[4]arene in the *trans* conformation of the azobenzene moiety but not for the *cis*-form, suggesting that the laser trapping of this azobenzene-based biscalix[4]arene is photo-controllable.^16^ The dynamics mechanism of the supramolecular assembly was considered, referring to the laser trapping-induced nucleation and liquid–liquid phase separation of amino acids (Fig. 3b).

**Fig. 3:** (a) The properties of amphiphilic photoresponsive gelators for aromatic solvents (4). (b) Photo-controlled supramolecular assembly of azobenzene-based biscalix[4]arenes (5).

The self-assembly of tris(phenylisoxazolyl)benzene (6) with photochemically addressable azobenzene moieties produced toroidal nanostructures, the formation, and dissociation of which were reversibly regulated upon photoirradiation. It displayed mesogenic behavior. In the solution, the stacked assemblies along with their *C*3 axes were formed. Two molecules of the antiparallel arrangement stabilized the columnar organization. This assembly behavior most likely triggered the development of the supramolecular toroidal nanostructures (Fig. 4a).^17^ However, an azobenzene-based mesogen (7) with a CN group at one end and a cholesterol carbonate attached to the opposite end was synthesized. It is a reversible photoresponsive chiral liquid crystal, capable of the formation of multi-stimuli-responsive organogels in organic solvents. The liquid crystalline, photoresponsive and gelling properties, as well as chiral induction and chiral amplification properties were demonstrated by different spectral techniques. It can act as a chiral mesogenic dye dopant to induce a highly helical twisting chiral phase in the common nematic phase of 5CB. This compound can show reversible photoresponsive properties in solution, in the liquid crystalline state, and the gel state. The gel formed by this compound in organic solvents can be reversibly modified under different environmental stimuli, including light, temperature, and shear. SEM and AFM revealed that the gelator molecules self-assemble into helical fibers of 58–130 nm in width and tens of micrometers in length, and these fibers form three-dimensional networks (Fig. 4b).^18^ The new series of azobenzene-based T-shaped asymmetric bolaamphiphiles (8) were synthesized, and their self-assembly behavior, photo-responsive behavior in their LC solution, and gel states were investigated. Such compounds can self-assemble into double-wall triangular and square honeycomb mesophases in their bulk states and organogels with different morphologies in various solvents. Irradiation of the gels with UV light generated gels with wrinkled structures. Co-assembly of these compounds with l-phenylalanine yielded organogels with helical structures. The influence of the azobenzene unit on the self-assembly behavior corresponded to self-assembly models (Fig. 4c).^19,20^ A barbiturate-functionalized supramolecular monomer (9) bearing an ester-linked biphenyl and azobenzene π-conjugated core afforded wavy supramolecular polymers. The periodic inversion of curvature is due to the conformational rigidity of the monomer and repulsive interactions between rosettes. Photoisomerization of the azobenzene moiety increases the fragility of the main chain without deteriorating its periodic structure (Fig. 4d).^21,22^

**Fig. 4:** (a) Photoresponsive toroidal nanostructure formed by the self-assembly of azobenzene-functionalized tris(phenylisoxazolyl)benzene (6). (b) Multistimuli responsive organogels based on a cholesterol–azobenzene dimesogen (7). (c) Asymmetric bolaamphiphiles of azobenzene (8). (d) Wavy supramolecular polymers were formed by hydrogen-bonded rosettes (9).

The photoresponse hydrogel (PR-gel) (10) was obtained by integrating 4arm-PEG and azobenzene into cellulose nanofibrils (CNFs). It has been proved to possess good mechanical strength, structural stability, and reversible recoverability. Benefiting from the introduction of the azobenzene cross-linker, the PR-gel also exhibited the reversible dynamic photochemistry isomerization transition originating from the *trans*–*cis* isomerism of azobenzene, and thereby caused a structural transformation and softening effect in its network, which could realize controllable BSA released by UV light irradiation. Good biocompatibility of the PR-gel was confirmed by the cell viability assay. The new insights into protein release vectors and cellulose-based stimulus-responsive hydrogels can help to expand the application fields of cellulose-based and some other sustainable materials (Fig. 5a).^23^ The formation of azobenzene-containing SCJNPs (11) occurred through the intrachain photo-crosslinking of linear PPEGMA-*b*-P(MAAz-*co*-MAStb) BCP precursors. The SCJNPs showed LC properties, as confirmed *via* DSC and POM studies. The self-assembly behavior of the resultant LC-SCJNPs in solution is quite different from that of the linear PPEGMA-*b*-P(MAAz-*co*-MAStb) BCP precursors. By adjusting the initial concentration and composition of the polymers, nonspherical self-assemblies, such as lamellae and tubes can be obtained facilely under the effects of the LC driving force. As the azobenzene moieties are tethered within the SCJNPs *via* intrachain cross-linking, the assemblies with higher azobenzene contents underwent reversible photoinduced deformation of the tube-connected spheres-tubes and spherical vesicles spheres-spherical vesicles upon exposure to alternating UV/vis irradiation. This work broadens the scope of self-assembly systems of SCJNPs and a reversible photoinduced morphology transition was achieved, in particular, a non-spherical morphological transition, which is of importance for many potential applications, such as functional materials and nanomedicines (Fig. 5b).^24^ Moreover, the UV light-triggered *trans*-to-*cis* isomerization of azobenzene (12) usually results in the collapse of a self-assembly system owing to the breaking of molecular planarity. Interestingly, two opposite self-assembly trends have been detected when a *C*_2v_-symmetric chiral gelator was irradiated by circularly polarized light (CPL) with specific handedness, indicating that CPL could become a powerful tool in modulating the assembly behavior of the photo-responsive system (Fig. 5c).^25^

**Fig. 5:** (a) Reversible photo-controlled release of bovine serum albumin by the azobenzene-containing cellulose nanofibrils-based hydrogel (10). (b) Self-assembly of single-chain Janus nanoparticles from azobenzene (11). (c) Supramolecular self-assembly of an azobenzene-based chiral gel (12).

## 3. Pyrene-based gel

The gelation properties of sugar–pyrene-based low molecular weight fluorescent gelators (13) show that the weak van der Waals interactions that exist between pyrene moieties are largely responsible for gelation. Functionalized SWCNTs did not show gelation properties due to the absence of weak interactions between the pyrene moieties. The interaction of SWCNTs with 13 had a negative effect on the gelation ability of the molecules. However, DSC studies showed that the functionalized SWCNTs and nanotubular gel had a greater thermal conductivity as compared to simple SWCNTs and pyrene-based gelators (Fig. 6a).^26^ In the photoluminescent pyrene-functionalized gelator (14), the excimer emission responds to thermo-reversible self-assembly. When the solvent matrix is polymerized around the gelator network, migration of the gelator leads to the accumulation of fluorescent gelator nanostructures at one face of the polymer wafer, giving rise to a ‘two-faced’ material. This approach to UV-controlled migration within a polymer matrix may be useful for controlling the photo-patterning of nanostructured materials (Fig. 6b).^27^

**Fig. 6:** (a) Fluorescent gelator of sugar–pyrene (13). (b) The structure of the ‘two-faced’ polymer–pyrene functionalized gelator nanofibres (14).

Non-amphiphilic pyrene cored poly(aryl ether) dendron derivatives (15) undergo solvent-controlled self-assembly in the system to result in nano-sized vesicles, which further aggregate into micro-sized vesicles and finally turn into an entangled fibrillar-type arrangement in the gel phase. The nano-sized vesicles and fiber aggregates exhibit intense light-emitting properties from the pyrene moiety attached to the dendron through an acyl hydrazone spacer group. Furthermore, the luminescence properties were found to be controlled by the solvent polarity, in a rather unusual manner, due to the selective formation of the pyrene ‘excimer’ and ‘exciplex’ in solvent-controlled aggregates. The system has been utilized to detect fluoride ions through a reversible gel–sol transition, which is associated with a color change from yellow to red (Fig. 7a).^28^ The multifunctional π-conjugated systems are derived from a renewable resource that self-assembles into supramolecular structures (16). The aggregation of compounds in different solvents strongly influences its optical properties. These π-conjugated molecules can be used for live-cell imaging applications. It also shows low cytotoxicity in fibroblast and suppresses the proliferation in PC_3_ prostate cancer cells (Fig. 7b).^29^

**Fig. 7:** (a) Non-amphiphilic pyrene cored poly(aryl ether) dendron-based gels (15). (b) Self-assembled π-conjugated system of pyrene (16).

A pyrene-based aminoquinoline-containing fluorescent probe 17 was investigated and the absorption and emission spectra revealed that the photophysical properties were significantly affected by the substitution of pyrene. It exhibited selective fluorescence behavior towards Zn^2+^ in aqueous solution. The gelation properties of these compounds were investigated by the “stable to inversion of a test tube” method. It displayed stable gel-formation properties in acetone, dioxane, tetrahydrofuran, ethyl acetate, chloroform, and dichloromethane. The xerogels were investigated *via* morphological studies. The temperature-variable ^1^H NMR spectroscopy suggested that both π–π stacking interactions and hydrogen bonding were the driving forces for the process of self-aggregation. It could form a stimuli-responsive gel that had a sensitive gel-to-sol transition response to heating and adding Zn^2+^ (Fig. 8a).^30^ In addition, two pyrene-functionalized gelator molecules 18 were designed, in which the pyrene moiety was directly linked to amphiphilic l-glutamide (PyC0) and with three methylene spacers (PyC3), respectively. They formed strong fluorescent organogels in polar and nonpolar solvents. Depending on the spacer, the pyrene gels showed different fluorescence. During the gel formation, the chirality in the l-glutamide moiety was transferred to the self-assembled nanostructures. While the PyC3 gels showed the same P-chirality in both the polar and nonpolar solvents, the PyC0 gel displayed chirality inversion in polar and non-polar solvents. It was suggested that the H-bonding between the amide groups and the π–π stacking between the pyrene moieties contributed to the formation of the gels, while the spacer between the amide groups and the pyrene ring regulated the two interactions, and thus influenced the assembly mode as well as the corresponding supramolecular chirality (Fig. 8b).^31^

**Fig. 8:** (a) Structure of the pyrene-containing fluorescent organogel (17). (b) Pyrene-functionalized organogel (18).

A fluorescent stimuli-responsive gel (19) was obtained from renewable resources by a simple process utilizing self-assembly. The hydrogen bonding and π–π stacking interactions that exist in the SG and MG stabilized the self-assembled structures. The morphological study depicted the formation of a highly entwined fibrous network with attached Fe_3_O_4_ nanoparticles. The stability and mechanical strength of SG and MG have been identified by rheological measurements. The magnetic properties and self-healing behavior of this system have been working well on the macroscopic level. SG and MG are both compatible for practical applications since they retained their inherent mechanical properties, even after processing the gels several times under different magnitudes of strain and temperature (Fig. 9a).^32^ The coumarin-coupled pyrene 20 with the varying hydrophobic units has been well characterized using NMR and mass spectral analysis. The self-aggregation properties of these compounds were studied relative to the molecular structure and solvent affinity. Among these derivatives, the one that does not have any hydrophobic tail displayed efficient gelation in higher alcohols such as decanol and dodecanol. However, the other derivatives having saturated and unsaturated hydrophobic tails form a weak gel in different solvents. The morphology of the gel was investigated by spectroscopy and microscopy techniques. The concentration-dependent emission and ^1^H NMR studies suggest the π–π stacking interactions and hydrogen bonding between carbonyl groups of coumarin coupled pyrene with the –OH groups of the solvent were the driving forces for the processes of gelation and self-aggregation. Rheological studies of the flow behavior and reversible nature of the organogel under temperature and strain ramp up and ramp down were conducted under experimental conditions. The size of the self-aggregated particles in the DMSO–water mixture has been identified using HRTEM and zeta sizer. The nanomaterials obtained *via* the self-assembly process have been used for fibroblast and PC_3_ prostate cancer cell imaging applications (Fig. 9b).^33^

**Fig. 9:** (a) Renewable resource-derived thixotropic self-assembled supramolecular gels (19). (b) Pyrene coupled coumarin derivatives of organogels (20).

Fluorescent glycolipids (21) were obtained from the direct condensation of vinyl esters with functionalized sugar alcohol using Novozyme 435, an immobilized lipase B from *Candida antarctica*. They were found to self-assemble into the gel in vegetable oils and highly hydrophobic solvents. A graphene-incorporated hybrid gel was also successfully obtained in linseed oil. The morphology of the gel was explored by optical microscopy and high-resolution transmission electron microscopy. The auto-oxidation of linseed oil present as a solvent in both self-assembled and graphene incorporated supramolecular gels resulted in the formation of flexible polymer films (Fig. 10a).^34^ The pyrene supramolecular gelator 22 is based on oxotriphenylhexanoate (OTHO), which can switch emission profiles between the solution and gel phase. A cocktail of the gelator and a photochromic diarylethene derivative enables four distinct emissive states to be obtained, which are modulated with light and heat as orthogonal input triggers (Fig. 10b).^35^

**Fig. 10:** (a) Gelation studies of fluorescent glycolipids (21). (b) Structure of the diarylethene pyrene–OTHO organogelator cocktail (22).

Pyrene-appended glucono-gelators (23) with different spacer lengths were found to form supramolecular gels in organic aqueous solvents. They are prone to self-assemble into nanotubes due to well-stacked multi-bilayer units. They show supramolecular chirality as well as circularly polarized luminescence (CPL) due to the chirality transfer from the glucose moiety to the assembly. The CD and CPL signals were opposite for the two gels. It was suggested that the packing of the pyrene unit in the gels was different due to the spacer and resulted in the inversed chiroptical properties (Fig. 11a).^36^ The pyrene-conjugated fluorescent organogels (24) have been examined by using various microscopic and spectroscopic techniques and rheological studies. Concentration-dependent fluorescence experiments show the excimer formation of gelator peptides in the aggregated gel state. This fluorescent organogel in ODCB is capable of incorporating unfunctionalized and non-oxidized graphene nanosheets into the organogel system by utilizing non-covalent π–π stacking interactions to form a stable hybrid organogel system. The hybrid organogel preserved the basic characteristics of the supramolecular gel, in particular, thermoreversibility and three-dimensional cross-linked nanofibrillar network structures. Rheological studies revealed that the storage modulus of the graphene-containing hybrid organogel is seven times more rigid than that of the native organogel. The construction of a graphene-containing hybrid fluorescent organogel system may open up interesting possibilities for the various nanotechnological applications of this type of graphene-based nanohybrid material (Fig. 11b).^37^ The morphology and mechanical properties of co-assembled gels (25) are dependent on the composition ratio of building blocks. The largest luminescence intensity of co-assembled gels was observed with a well-organized molecular arrangement of excimers. The morphology of the co-assembled supramolecular gels changed from spherical nanoparticles to three-dimensional network nanofibers. Thus, further development of co-assembly supramolecular gels using the formation of pyrene-excimer can offer materials for optical applications and dual-functional gels by implementing functional derivatives (Fig. 11c).^38^

**Fig. 11:** (a) Self-assembly of pyrene-appended glucono-gelators (23). (b) Pyrene containing peptide-based fluorescent organogel (24). (c) Pyrene-based co-assembled supramolecular gel (25).

The pyrene derivatives (26) were determined by density functional theory (DFT) calculations. The results of photophysical spectra and electrochemical analysis indicated that the optical and electric properties of the pyrene derivatives could be tuned by adjusting the π-conjugation lengths of the substituents. Furthermore, through a phase exchange self-assembly method, the highly organized morphologies were observed by SEM (Fig. 12a).^39^ Moreover, the 1,2,3-trioctyloxyphenyl-based organogel (27) can form stable organogels with dramatic aggregation-induced emission (AIE) in some organic solvents. It was investigated *via* concentration-dependent studies using ^1^H NMR, XRD, FT-IR, and SEM techniques. In addition, it shows good fluorescence sensing ability to some anions such as F^−^ and AcO^−^. In DMF solution, the addition of F^−^ to the organogel showed a gel–gel phase change with quenched AIE. However, the addition of AcO^−^ led to a gel–sol transition with few fluorescence changes (Fig. 12b).^40^ The fluorescent gelator (28) was synthesized, which efficiently gelatinized the aqueous medium. This was revealed through different spectroscopic and microscopic techniques. Diverse functions of the gelator have been observed including potential applications in the development of gel-nanoparticle soft composites. AgNPs were synthesized *in situ* within the hydrogel by exploiting the free amine (–NH_2_) group of amphiphiles at ambient temperature under sunlight. These AgNP soft nanocomposites could find potential applications in the development of antibacterial soft materials because of the inherent bactericidal effects of AgNPs (Fig. 12c).^41^

**Fig. 12:** (a) Self-assembly properties of asymmetrical pyrene derivatives (26). (b) Structure of pyrenyl-appended organogel (27). (c) Pyrene-based fluorescent supramolecular hydrogel (28).

The ambidextrous gelator (29) was an efficiently gelatinized organic solvent as well as aqueous media at suitable pH. The crucial role of the HLB in self-assembled gelation was studied by the sensible alteration of the amino acid residue present in the gelator. The mechanism of gelation by the involvement of different supramolecular interactions has been illustrated through spectroscopic and microscopic studies. SWNTs can be successfully incorporated into both the hydro- and organogel matrices of the synthesized AGs to produce stable SWNT-gel nanohybrids. Furthermore, the fluorescent nature of the native gels and SWNT-included nanohybrids should find immense importance in the field of materials science, as well as in biomedicinal applications (Fig. 13a).^42^ A modular molecule (30) constituted a multipolar D–π–A unit, H-bonding groups, encapsulating unit, chiral centers, and fluorophore units. The molecule crystallizes in one of the ten polar point groups, satisfying the symmetry prerequisites for some important material properties such as NLO, ferroelectricity, and piezoelectricity, which are characteristic of this molecule in the solid-state (Fig. 13b).^43^ Bis-pyrene (BP) (31) can self-assemble into a highly-ordered columnar mesophase structure. On the other hand, BP can self-assemble into nanofibers in solution. More importantly, BP showed interesting dually controllable quenching and emission fluorescence in solvent, which is an AIE phenomenon (Fig. 13c).^44–48^

**Fig. 13:** (a) Pyrene-based fluorescent ambidextrous gelator (29). (b) Self-assembly characteristics of bis-pyrene (30). (c) Unique fluorescence properties of a self-assembling bis-pyrene molecule (31).

## 4. Perlylene-based gel

The agglomeration of self-assembled fibers of p-conjugated molecules is crucial to the formation of low-molecular-weight supramolecular gels (32). However, the identification of the *in situ* spectroscopic signatures of fiber agglomeration has remained a challenging endeavor. A combination of chiroptical techniques was used to investigate the agglomeration of self-assembled fibers of a chiral low-molecular-weight gelator, l-alanine-substituted perylene imide bis(*n*-butyl) ester (PIBE). Remarkably, agglomerated PIBE fibers exhibit the opposite CD signature in comparison to the isolated PIBE fibers. In contrast, the MCD and FDCD responses do not change during the agglomeration process, revealing that the local structure in the individual fibers is unperturbed. Using Brownian dynamics simulations, the effective charge on the fibers dictates the agglomeration process, and the final geometry of the agglomerated fibers is marked by crossed nodes (Fig. 14a).^49^ Moreover, the amino acid–PBIs (33) can form one-dimensional structures at high pH and then gels at low pH. Both the dried solutions and dried gels are photoconductive. Remarkably, the photoconductivity of these materials requires that the incident light has a wavelength shorter than 400 nm, in stark contrast to the absorption maxima of the PBIs. The photoconductivity correlates with the formation of the perylene radical anion, which is unusually highly stable in air for many hours (Fig. 14b).^50^ There was an unexpected formation of PBI dye (35) aggregates with strongly bathochromically shifted J-type absorption bands in solution. The organogel state was from core-unsubstituted PBIs upon the subtle variation of the peripheral alkyl side chains. The combination of intense absorbance over the whole visible range led to a dark green to almost black color and the ability to form defined extended supramolecular networks in various kinds of organic media, which provides unique possibilities for these materials as photosensory systems or as n-type semiconductors in organic bulk heterojunction solar cells (Fig. 14c).^51^

**Fig. 14:** (a) The formation of perylene-based fiber networks (32). (b) Air-stable photoconductive films formed from perylene bisimide gelators (33). (c) Structure of the perylene bisimide super gelator (34).

The perylene-based hydrogels (35) were formed spontaneously upon mixing a simple perylene diimide derivative with melamine. These gels exhibit highly intense fluorescence visible to the naked eye. The resulting gel network consists of the inner core of H-stacked perylenes cross-linked by MMs and a water-soluble carboxylic acid at the outer surface. The perylene derivative forms a gel in the aqueous medium (Fig. 15a).^52^ Organogels with perylene derivatives (36) involve self-assembly promoted by hydrogen bonds, in addition to aromatic and van der Waals interactions. The self-assembly of these types of molecules without a hydrogen-bonding group in the structure occurs in solution or during crystallization. The gelation studies reported so far incorporated a hydrogen bonding pair of the type [N–H/O]C in the structure of the molecule. The PDMS segment was attached to one side of PDI (mono-PDMS) or both imide nitrogens of PTCDI (di-PDMS). The mono-PDMS is an inverse macromolecular surfactant applicable to non-aqueous systems, and the di-PDMS is a Gemini surfactant. The PDMS segment that we attached to PTCDI is longer than most substituents used by other authors. These molecules gel propylamine, as well as mixed solvents of hexane–water and diisopropylamine–water. Both hexane and diisopropylamine dissolve mono-PDMS and di-PDMS at room temperature and the addition of water results in precipitation. Although the mono-PDMS and di-PDMS are a homologous pair, blends of these do not show molecular intercalation during gelation. The fibers of di-PDMS-based gels encapsulate the spheres of the mono-PDMS-based gels (Fig. 15b).^53^ Recognition-directed spontaneous assembly formation has been used to build up a sensory system with perylene bis-guanidinium (37), which presented a great response toward chiral guest sensing. It can selectively recognize dibenzoyl tartaric acid, and DBTA among other tartaric acids (TA), resulting in an explicit read-out of the molecular information *via* the generation of the characteristic induced circular dichroism spectra for d- and l-enantiomers. The binding ability depends only on the substituents in the TA, and the local guidances play an important role in structure formation. The bulky substituents in TA can induce chirality into the cofacial perylene stacks by generating an active angle between the successive transition dipoles. The induced helical sense was found to exhibit efficient chiral amplification with a sigmoidal change in the enantiomeric excess plot. The diversity in physical properties was further entertained by the preparative method, and the heating-cooling method, compared to the simple mixing method. It can show aggregation-induced fluorescence enhancement, which was used to fabricate a highly efficient fluorescent solid in a supramolecular manner, even from a perylene-based dye (Fig. 15c).^54^ Supramolecular gels from l-aspartic acid-based perylene bisimides (APBI) and various isomeric benzene dicarboxylic acids were obtained. It has been found that the spatial position of carboxyl on the benzene ring plays a key role in the gelation process. Intermolecular hydrogen bonding has been found to guide the aggregation determined by FT-IR. The interesting features of the two-component gel system may give a better understanding of supramolecular chirality (Fig. 15d).^55^

**Fig. 15:** (a) Assemblies of perylene diimide derivatives with melamine into luminescent hydrogels (35). (b) Thermo-reversible gelation of rod-coil perylene imides (36). (c) Molecular recognition of perylene–bisimide aggregation (37). (d) Formation of supramolecular chiral gels (38).

The co-assembly of achiral PBI with chiral gelators (39) can be regulated by ethanol and an acid–base responsive CPL switch. Avoiding tedious organic synthesis and purification, the supramolecular cogelation of a chiral gelator and achiral dye affords a new approach for fabricating CPL-active gel materials. By selecting the appropriate solvent, cogel formation could enable chirality transfer from the chiral gel to the achiral dye. An acid–base fumigation-driven CPL switch could be realized based on both chirality transfer and reversible protonation of the cogel (Fig. 16a).^56^ Moreover, the amino acid-functionalized perylene bisimides (PBIs) (40) affected the self-assembled aggregates and resulted in physical and optical properties. PBIs functionalized with l-valine (PBI-V), l-leucine (PBI-L), and l-isoleucine (PBI-I) were investigated due to their similarly branched structures and their assemblies in water were studied using spectral techniques. It was seen that each PBI behaved differently. They were then used to prepare hydrogels, and their properties were again assessed, with PBI-I forming different hydrogels than the other PBIs (Fig. 16b).^57^ In addition, the PBI-based organogel systems (41) were obtained by melamine–melamine, melamine–cyanurate, and melamine–barbiturate multiple hydrogen-bonding interactions. The gelation capability of these systems is based on the number of chromophore units in melamine molecules. They were transparent and showed remarkably low critical gelation concentration. XRD studies revealed that the gelation of solvents was caused by the hierarchical organization of tape-like hydrogen-bonded aggregates. However, the mesoscopic structures of the aggregates observed by SEM and AFM were different, depending on the number of the PBI chromophores in the melamine components. As a result, the gels showed different thermal stabilities. It is proposed that the number of the PBI chromophores introduced in the melamine components can control the hierarchical organization process of the tapelike hydrogen-bonded aggregates (Fig. 16c).^58^ A series of LC perylene bisimides (PBIs) (42) were self-assembled into single or multi-stranded aggregates with predominant J-type exciton coupling. These differences in the supramolecular packing and optical properties were achieved by molecular design variations of tetra-bay phenoxy-dendronized PBIs with two –NH groups at the imide positions. The self-assembly is driven by hydrogen bonding, slipped π–π stacking, and steric requirements of the peripheral building blocks. The impact of the packing motifs on the spectroscopic properties demonstrates different J- and H-type coupling contributions between the chromophores (Fig. 16d).^59^

**Fig. 16:** (a) Co-assemblies of the chiral gelator with achiral perylene bisimide (39). (b) Self-assembly of perylene bisimides hydrogels (40). (c) Structure of perylene bisimide organogels (41). (d) Self-assembly of multi-stranded perylene dye (42).

Two-component hydrogels (43) with networks composed of self-sorted fibers are based on 1,4-distyrylbenzene (OPV3) and perylene bisimide (PBI) units. They can be formed by a slow decrease in pH, which leads to sequential assembly. Photoconductive xerogels can be prepared by drying these gels. The wavelength response of the xerogel is different from that of the PBI alone (Fig. 17a).^60^ A stable organogelator (44) containing perylene bisimide–aminocaproic acid and imidazole units, which was linked by strong hydrogen bonding interactions, was successfully designed and characterized. It was able to form fluorescent organogels in DMSO either by a heating-cooling process or ultrasound treatment *via* π–π stacking, hydrogen bonding, and hydrophobic interactions. The obtained gels exhibited fluorescence enhancement characteristics. It was proposed that the inhibition of fluorophore aggregation, ordered arrangement of molecular aggregations in fibers, as well as reduction of radicals, were all important for fluorescence enhancement in 3D gel networks (Fig. 17b).^61–64^

**Fig. 17:** (a) Self-sorted perylene bisimide hydrogels (43). (b) Emission enhancement of the perylene–bisimide-based organogel (44).

## 5. Coumarin-based gel

A photocleavable low-molecular-weight hydrogelator (LMWG) was synthesized based on a coumarin derivative (45). ^1^H NMR and UV spectroscopy studies suggested that the gelator had good gelling ability, and the driving force for the gelation was hydrogen bonding and π–π stacking. It exhibited satisfactory photocleavage at the C–N bond in 7-aminocoumarin with light irradiation. The photo-triggered drug release of antineoplastics cytarabine hydrochloride was obtained, due to the photocleavage-motivated gel–sol transition (Fig. 18a).^65^ Moreover, the two 3-styryl coumarin molecular rotors (46) are capable of probing subtle intermolecular interactions controlling the self-assembly of a small-molecule organogelator. To complement the characterization of the gel *via* circular dichroism and atomic force microscopy, thorough spectroscopic investigations on these sensors were carried out to prove their high chemical and spatial affinity toward the 3D supramolecular network. The results were further supported by molecular dynamics simulations to reveal further critical insights into the gelator's dynamic self-assembly mechanism. These sensors could potentially serve as templates to study a variety of soft supramolecular architectures (Fig. 18b).^66^

**Fig. 18:** (a) Photo-cleavable low molecular weight hydrogel (45). (b) Photophysical behavior of coumarin (46).

A redox-responsive chiral supramolecular gel was obtained based on coumarin-tailed cholesterol linked with disulphide (47), primarily driven by the combination of hydrogen bonding, π–π stacking, and van der Waals forces. The gel morphology could be regulated by water from nanofibers to microflowers and microribbons on account of its amphiphilic characteristics. Moreover, the supramolecular gel exhibited excellent redox-responsive properties, which may be used in controlled release and drug delivery (Fig. 19a).^67^ In addition, the coumarin-appended 1,2,3-triazole-coupled cholesterol (48) has been designed and synthesized, which acts as a small molecular gelator. It has been noted to form a gel from CHCl_3_–petroleum ether. The stable gel is anion-responsive. The gel state is transformed into the sol state selectively in the presence of F^−^ and hydrogen pyrophosphate, which validates its visual sensing over a series of other anions. Fluorescence studies in CH_3_CN containing 0.5% DMSO also revealed the substantial change in emission of 48 upon the addition of both F- and hydrogen pyrophosphate and distinguished them from other anions studied (Fig. 19b).^68^

**Fig. 19:** (a) Redox-responsive behavior of the supramolecular gel (47). (b) The structure of the coumarin-based supramolecular gelator (48).

The coumarin-based dipeptide gelator (49) can form hydrogels using a pH switch using both GdL and hydroquinone. The gels can photodimerise after irradiation with a 365 nm LED. This irradiation leads to an increase in the rheological properties, which is believed to be caused by the dimerization within fibers stiffening them, rather than cross-linking being formed between fibers. This opens up the possibilities of enhancing the gels post-gelation, or locking in a structure by covalent dimerization. The use of UV light could also be used to photo-pattern surfaces for applications such as cell culture and differentiation (Fig. 20a).^69–73^ The tetrapeptide–coumarin conjugate (GVGV–Cou) (50) has been investigated along with its ability to encapsulate and release guest molecules. Anti-parallel β-sheets can be formed between peptide segments *via* the formation of H-bonds. The formation of such a strong CT complex might be facilitated by the strong ability of the GVGV peptides to form β-sheets. Based on the collaborative interactions of hydrogen bonding and CT interaction, GVGV–Cou was assembled into a stable gel composed of fibrous structures. Furthermore, the gel can be used as a matrix for the encapsulation and release of dye molecules (Fig. 20b).^74^

**Fig. 20:** (a) Photodimerisation of a coumarin–dipeptide gelator (49). (b) Tetrapeptide–coumarin conjugate of 3D networks (50).

A multi-functional gelator precursor (51) with high photosensitivity was rationally designed, which can selectively target cancer cells through the receptor-mediated interaction between galactose and ASGP-R overexpressed by cancer cells. It can release hydrogelators inside cells under photo-irradiation, leading to intracellular self-assembly, subsequently inducing cell death. They have the property of two-photon absorption, enabling the irradiation of the precursors with near-infrared light. Multi-functional nano-materials for selective and efficient tumor therapeutics can be realized by precisely releasing the assembled gelators under external stimuli. They can be further exploited in the design of similar systems to target different cancer cells by exchanging the galactose unit with other functional groups, which can specifically recognize the receptors over-expressed at the cell membrane (Fig. 21a).^75^ Furthermore, the coumarin chromophores (52) have been combined into the rigid core of polycatenars with two triazole wings to yield hexagonal LCs with different 2D columnar phases and gels with complex morphologies. They can be extended to LC and gel states as established carefully by spectroscopy techniques. The nanostructures of the mesophases and microstructures of the gels were studied in detail by POM, DSC, XRD, and SEM. The reversible photodimerization of coumarin polycatenars in both LC and gel phases proceeded with an interesting change in both LC phase structures and gel morphologies (Fig. 21b).^76^

**Fig. 21:** (a) Light-responsiveness of the galactose-decorated hydrogelator (51). (b) Structure of coumarin-based emissive hexacatenars (52).

The acyl hydrazone-based coumarin derivative gelator (53) was formed as a supramolecular polymer gel OGC *via* π–π stacking, van der Waals, and intramolecular hydrogen bonding. OGC showed green-yellow AIE fluorescence in *n*-EtOH/H_2_O binary solution and could successively detect and separate toxic ions in the gel state with high selectivity and sensitivity. Thin films based on the supramolecular polymer gel OGC were prepared, which were confirmed to be convenient thin films for sequentially detecting CN^−^, Fe^3+^ and S^2−^, Ag^+^. An efficient method for the development of supramolecular polymer gels to detect toxic ions is the construction of supramolecular systems (Fig. 22a).^77^ A coumarin-derived acyl hydrazone Schiff base fluorescent organogel (54) can form stable organogels in isopropanol, *tert*-amyl alcohol, *n*-butanol, and phenylamine. It can respond to heating, irradiation, and vigorous agitation, and the solution can be reformed to the gel state after being cooled for about 0.5 h. The supramolecular aggregation in solution was investigated through concentration *via* spectroscopic studies. All the results indicated that the hydrophobic interactions between alkyl chains, the π–π stacking interactions between the coumarin moieties, and the hydrogen bonding between the acyl hydrazone/Schiff base moieties play important roles during the formation of ordered gels. Metal cation selectivity studies with the gel factor Fe^3+^ complex in the fluorescence spectroscopy revealed that the complex is easily detected in the presence of the Fe^3+^ (Fig. 22b).^78^

**Fig. 22:** (a) Supramolecular polymer gel-based long-alkyl-chain-functionalized coumarin (53). (b) Schiff base-based coumarin gelator (54).

The series of 1,2,3-triazoles functionalized with coumarin (55) are efficient gelators while the hydrogenous-triazole exhibit no gelling efficiency. The existence of an iodine atom in the 5-position of the triazole ring is vital to the gelating ability of the compound. It shows a response to mercury ions and can conduct reversible photodimerization. The morphology of the gel changes prominently under irradiation at 365 nm light and it can partly recover after the subsequent exposure to 254 nm light. Plots were constructed to show the gelation behavior of the gelator in pure solvents and mixed solvents (Fig. 23a).^79^ A new kind of coumarin-based photoresponsive hydrogelator DPC (56) can self-assemble into nanofibrous structures in an aqueous solution. The resulting DPC hydrogel can be disintegrated due to the photomediated cleavage of the DPC gelators under UV light irradiation, resulting in the precise and efficient release of encapsulated agents. Such controllable disassembly of hydrogel networks leads to the great potential of soft materials for controlled drug release under external stimuli (Fig. 23b).^80^ Photoinduced reinforcement of supramolecular gel structures (57) has been achieved using photodimerization of coumarin moieties introduced into gelator molecules. The photodimerization reaction in the self-assembled fibers of gelators enabled the enhancement of both the thermal and mechanical stabilities of the gels. There is still room for improvement to achieve efficient and reversible reinforcement due to the limitation of the gelation solvents and the low content of coumarin moieties (Fig. 23c).^81^

**Fig. 23:** (a) Organogelators based on iodo 1,2,3-triazole functionalized with coumarin (55). (b) Photoresponse of the coumarin-based supramolecular hydrogel (56). (c) Photoinduced reinforcement of supramolecular gels (57).

## 6. Rhodamine-based gel

2,6-Diaminopyridine-coupled rhodamines (58) have demonstrated the effect of substitution on amine functionality toward metal-ion interactions. The compounds effectively recognize different metal ions of biological significance fluorimetrically and colorimetrically with a high degree of selectivity and sensitivities. The sensing mechanism involves the metal-ion chelation-induced spirolactam ring-opening of the rhodamine scaffold that results in both color and fluorescence changes, while the extent of interactions with the metal ions is truly governed by the chemical structure of the compounds. They are proficient in detecting Fe^3+^ and Al^3+^ ions in human lung cancer cells (Fig. 24a).^82^ The rhodamine-based *N*-glycosylamines (59) were characterized using different spectral techniques. They act as good organogelators and can gelate even at a CGC of 1 w/v%. Morphological, thermal, and powder XRD studies show the various modes of aggregation and stability of gels, respectively, which depend on the protecting groups and also on the substituents in the rhodamine moiety (Fig. 24b).^83^ A 3-aminomethyl-(2-amino-1-pyridyl) coupled amino-ethyl-rhodamine-B-based probe (60) exhibited simultaneous fluorogenic dual mode signaling responses in the presence of Hg(ii) ions only among all the metal ions investigated in an organic aqueous medium. The spiro-cyclic rhodamine signaling subunit underwent complexation-induced structural transformation to result in absorption and fluorescence modulation. Its complexation-induced signaling exhibited reversibility with various contrasting reagents having a higher affinity towards Hg(ii) ions. It also exhibited Hg(ii)-specific photophysical signaling responses when immobilized on a silica gel surface attached through its amino-ethyl-receptor end, owing to its structure-conformational advantages for effective coordination. The surface-modified silica appended with (SiR-1) exhibited reversible Hg(ii)-specific signaling in its suspension state in aqueous medium. The probe can be utilized for practical applications such as the detection, isolation, and extraction of Hg(ii) ions in the presence of other competitive metal ions (Fig. 24c).^84^ Moreover, a reversible solid optical sensor (SGIR) for Hg^2+^ based on silica gel (61) was designed and synthesized. The binding and adsorption abilities of SGIR for metal cations were investigated with fluorophotometry and cold vapor atomic absorption spectrometry, respectively. It exhibited high selectivity for sensing Hg^2+^ over other metal cations in aqueous media because the Hg^2+^ ion selectively induces a ring-opening of the rhodamine fluorophores. The determination of Hg^2+^ in both tap and lake water samples displayed satisfactory results and the SGIR can also be easily recovered by treatment with a solution of TBA^+^ OH^−^ (Fig. 24d).^85^

**Fig. 24:** (a) 2,6-Diaminopyridine-coupled rhodamine in metal-ion interactions of self-assembly (58). (b) Gelation studies of rhodamine-based *N*-glycosylamines (59). (c) Dual-mode signaling responses of a rhodamine-based probe (60). (d) Dual functional of rhodamine-immobilized silica (61).

A new hybrid PVOH film bearing a rhodamine derivative ligand (62) was used as a naked eye colorimetric sensor for the detection of Fe^3+^ ions in aqueous systems. It exhibited excellent selectivity and sensitivity toward Fe^3+^ ions over a wide range of metal ions *via* an emerging UV-vis absorption peak at 556 nm and an obvious visible change in the solution color to pink. Then, this molecular chemosensor was covalently coupled to the crosslinked PVOH films by a sol–gel process. According to Job's plot, the proposed sensing mechanism was described by a 1 : 1 binding stoichiometry. The Fe^3+^ ion sensing of the hybrid chemosensor was reversible and the chemosensor could be reused several times without significant signal reduction (Fig. 25a).^86^ Moreover, a fluorescent nanofibrous hydrogel (63) for long-term cell tracking and tumor imaging applications can be obtained by dilution of the hydrogel with an aqueous solution. The resultant nanofibers with low cytotoxicity can effectively trace the HeLa cells for as long as 7 passages. The *in vivo* studies revealed that as compared to the precursor, the nanofibers can preferentially accumulate in tumor tissues by the EPR effect, allowing for tumor imaging in a high-contrast manner. The red fluorescence allows the nanofibers to be used for bioimaging applications due to the relatively low interferential absorption and relatively high tissue penetration (Fig. 25b).^87^ The multi-functional rhodamine-based chitosan hydrogels (64) demonstrated sensing properties through the incorporation of fluorophores. Strong valency forces were formed between the active N/O atoms and Hg^2+^ through the sharing of lone pair electrons, resulting in the chelation of the RMC hydrogel towards Hg^2+^ with fluorescence enhancement. The sensitivity of the hydrogel was due to adsorbents with functional fluorophores, which may be achieved through adjusting the molecular structure or aggregation state of the fluorophores in hydrogels. More eco-friendly bio-sorbents with low biotoxicity and high mechanical strength should be developed for industrial applications (Fig. 25c).^88,89^

**Fig. 25:** (a) The sol–gel technique for the selective detection of Fe^3+^ ions (62). (b) Biocompatibility with the fluorescent supramolecular nanofibrous hydrogel (63). (c) Multi-functionality of rhodamine-based chitosan hydrogels (64).

A summary of selected types of fluorophores, gel structures, and applications referenced is given in Table 1 below.

**Table 1:** Summary of types of fluorophores and associated gel structures involved in this review

Types of fluorophores	Types of gel structures	Applications	Ref.
Azobenzene–cholesterol	Organogel	—	11
Azobenzene–phenylalanine	Supramolecular gel	Adsorption	12
Azobenzene–sugar	Organogel	—	13–15
Azobenzene biscalix[4]arene	Supramolecular gel	—	16
Sugar–pyrene	Fluorescent gel	Functionalized SWCNTs	26
Pyrene–aminoquinoline	Organogel	Fluorescent probe	30
Coumarin coupled pyrene	Organogel	PC_3_ prostate cancer cell imaging	33
Perylene bisimide–aminocaproic acid and imidazole units	Organogel	3D gel networks	61–64
Coumarin-tailed cholesterol	Supramolecular gel	Drug delivery	67
Coumarin–dipeptide	Hydrogel	Cell culture	69
Rhodamine–chitosan	Hydrogel	Bio-sorbents	88

## 7. Conclusion

Herein, we have summarised gel scaffolds and their emerging applications in biomedicine-related applications. These include hydrophilic biomaterials, and some commercially accessible hydrogel materials that have been approved for use in biomedicine. The processability and optical clarity of hydrogels have paved the way for optical applications. The addition of luminous matter to functional hydrogel scaffolds is an intriguing extension. They have established themselves as a bridge platform for fluorescence-based applications in health care, such as sensing, imaging, and actuation.

## Conflicts of interest

There are no conflicts to declare.

## Abbreviations

NMR: Nuclear magnetic resonance
DSC: Differential scanning calorimetry
SEM: Scanning electron microscope
AZO-Phe: Azobenzene phenylalanine
MB: Methylene blue
AFM: Atomic force microscopy
UV: Ultraviolet
CNFs: Cellulose nanofibrils
PR-gel: Photoresponse gel
CPL: Circularly polarized light
HRTEM: High-resolution transmission electron microscopy
DMSO: Dimethylsulfoxide
OTHO: Oxotriphenylhexanoate
DFT: Density functional theory
AIE: Aggregation induced emission
DMF: Dimethylformamide
XRD: X-ray diffraction
BP: Bis-pyrene
PIBE: Perylene imide bis(*n*-butyl) ester
DBTA: Dibenzoyl tartaric acid
TA: Tartaric acids
LMWG: Low molecular weight gelator
CHCl_3_: Chloroform
CH_3_CN: Acetonitrile
Hg: Mercury
CGC: Critical gelation concentration

## Supplementary Material
